# A Study on the Optimization and Improvement of the Construction of the Campus Football Development Model by a Factor Analysis Method under the Background of “Healthy China”

**DOI:** 10.1155/2022/3260571

**Published:** 2022-05-26

**Authors:** Zhen Wang, Bin Tan, Binquan Yi

**Affiliations:** School of Physical Education, Hunan Institute of Science and Technology, Yueyang 414006, China

## Abstract

In order to enrich campus sport life and promote the development of campus ball game, this paper uses the analysis method to analyze the development mode of campus football and evaluates the relevant factors combined with the development status, characteristics, and future trend of campus football. Factor analysis is a comprehensive analysis method, which can realize multifactor comprehensive analysis and qualitative and quantitative analysis of campus football. At the same time, analyze the relationship between various factors and find a scheme conducive to the development of campus football. The results show that both comprehensive method factors and single method factors are positive, indicating that the two models have a significant positive impact on the development model of students' football. However, the influence degree of the comprehensive method (0.314) is the largest, followed by the single method factor (0.128), and the sig. values of the two variable factors are <0.05, so the comprehensive method is the main mode of campus football development. Therefore, the factor analysis method proposed in this paper is conducive to the selection of campus football development model and provides support for the development of campus football.

## 1. Introduction

At present, the development of campus football in China is divided into four modes: single football mode, mixed development mode, learning from foreign modes, and self-innovation mode, each accounting for 7%, 10%, 26%, and 57%, respectively. Among them, mixed development and foreign models are comprehensive methods, while self-innovation and single football model is single methods. However, the results of different development models are different so that colleges and universities cannot choose their own campus football development model. Factor analysis is to use a few factors to describe the multiple indicators affecting the campus football model and determine the relationship between different factors. Factor analysis is to use a few factors to describe the multiple indicators affecting the campus football model (Brahmachary et al.) [1] and determine the relationship between different factors. Factor analysis method uses cluster analysis to classify the variables with high correlation into the same category, and each category of variables becomes a factor, which reflects most of the information of the original data through fewer factors [2]. Because the factor analysis method has its own shortcomings, it cannot realize the analysis of massive data and dynamic data, so it is necessary to combine the correlation function to make up for the shortcomings of its own analysis. Therefore, the development process of campus football is complex and involves many factors. How to better analyze and improve the accuracy of analysis results is an urgent problem to be solved at present. Factor analysis has comprehensive characteristics, which makes each influencing factor dynamic and standardized, and makes better analysis. Factor analysis can easily find out the main factors affecting the development mode of campus football and the influence of each factor so as to realize the comprehensive analysis of campus football. Content of campus football⟶Influencing factors of campus football⟶Factors of campus football⟶Determine the main factors of campus football⟶Construct a series diagram of impact factors⟶Make an impact factor map. Taking campus football as the research object, this paper studies the relationship between each factor and the development model of campus football through multifactor analysis of the development model.

## 2. Literature Review

Factor analysis has more research on ball games, but less research on football development model. Some scholars believed that football is affected by many factors such as age, gender, and region [3]. It needs to choose the development model in combination with different objective conditions [4]. In addition, different development models have different effects on football, so we should make a comprehensive analysis of multiple factors with the help of qualitative and quantitative analysis methods. Some scholars believed that the amount of data of campus football was small, and historical data cannot be used for analysis [5], so it was not suitable for large-scale statistical analysis. Some scholars also put forward eigenvalue analysis methods, which used a small amount of confirmed value data to carry out relevant analysis and research, and reflected the overall data characteristics, such as factor analysis method, the decision tree method, etc. [6]. To sum up, scholars at home and abroad had unified opinions on the development model of campus football and believed that the development model of campus football should be combined with its own situation for comprehensive and comprehensive analysis [7]. However, there are many problems in campus football, such as less data and more influencing factors [8]. Therefore, factor analysis and the analytic hierarchy process are suitable analysis methods.

## 3. Relevant Models

### 3.1. Overview of Factor Analysis

Factor analysis, as a comprehensive analysis method, mainly analyzes various factors and indicators comprehensively, and studies the influence degree of each factor on the final result. Finally, factor analysis determines the main factors in the analysis results and the role played by this factor. According to the results of factor analysis, some opinions and suggestions are put forward. Compared with other analysis methods, the results of factor analysis are more objective and accurate.

### 3.2. Mathematical Descriptions of Football Development Model

Assuming that any football pattern *x*_*i*_ is a observable random vector and its set is {*x*_1_,…, *x*_*n*_}, the vector formula is Ex(*x*), the covariance matrix is Co(*x*), and the factor calculation formula of different vectors is shown as follows [9]:

(1) $$\begin{array}{c} \text{Co}\left(x\right)=\frac{\sum_{i=1}^{n}x_{i}}{Ex\left(x_{i}\right)}+\xi , \end{array}$$

where *ξ* is the adjustment error of the factor. Assuming that the correlation of any football pattern is *f*_*j*_, which is a random observable vector and its set is {*y*_1_,…, *y*_*m*_}, the vector formula is *F*(*x*), the covariance diagonal matrix is *E*(*x*)=Σ, and the correlation calculation formula of different factors is shown as follows:

(2) $$\begin{array}{c} E\left(y_{i}\right)=\frac{\sum_{j=1}^{n}x_{j}}{F\left(x_{j}\right)}+\tau , \end{array}$$

where *τ* is the adjustment error of correlation [10]. The mode selection formula of factor analysis method is constructed according to formulas (1) and (2), and the results formula is shown as follows:

(3) $$\begin{array}{c} y_{j}=\text{Co}x\left(x_{i}\right)+E\left(y_{i}\right)+\xi +\tau . \end{array}$$

In order to improve the accuracy of the calculation results, it is necessary to construct the influencing factor matrix to realize the comprehensive analysis of the development mode of campus football. The specific calculation formula is shown as follows [10]:

(4) $$\begin{array}{c} y_{j}=\left[\text{Co}x\left(x_{i}\right)+E\left(y_{i}\right)+\xi +\tau \right]\cdot \left(\begin{array}{ccc} z_{11} & \ldots & z_{1n}\\ \vdots & \ddots & \vdots \\ z_{m1} & \ldots & z_{mn} \end{array}\right), \end{array}$$

where $\left(\begin{array}{ccc} z_{11} & \ldots & z_{1n}\\ \vdots & \ddots & \vdots \\ z_{m1} & \ldots & z_{mn} \end{array}\right)$ is the influencing factor judgment matrix and${\left(\begin{array}{ccc} z_{11} & \ldots & z_{1n}\\ \vdots & \ddots & \vdots \\ z_{m1} & \ldots & z_{mn} \end{array}\right)}^{T}\neq 0$.

### 3.3. Research Assumptions

Based on previous studies, this paper puts forward relevant basic assumptions H_1_, H_2_, and H_3_. In the empirical analysis, variance and correlation analysis is used to verify the relevant basic assumptions [11]. After verification, most of the assumptions are true or partially true. The result is shown in Table 1.

### 3.4. Variable Designs and Model Construction

Firstly, project preparation was performed. This paper combines the interview results and open-ended questionnaire survey results, including demographic characteristics survey, such as gender, age, experience, and so on. The second part is the evaluation effect of corresponding indicators, which is composed of 1–5 points, representing nonconformance, basic conformance, conformance, relatively conformance, and very conformance [12]. Secondly, the reliability analysis is the reliability analysis of the effect questionnaire, in which the values of each variable and factor *α* are shown in Table 2.

According to Table 2, the overall reliability of the campus football development model measurement table is 0.835, which is at a high reliability level.

#### 3.4.1. Validity Analysis

This paper uses the KMO test and Bartlett's sphere test to analyze the survey data so as to determine whether the items in the questionnaire meet the effect of factor analysis. The result is shown in Table 3.

The KMO value is 0.826, DF (degree of freedom) is 27, Sig. < 0.01, which has significant difference, representing the suitability for factor analysis. After Bartlett's spherical test, this questionnaire obtains a significant chi-square value, which further shows that it is suitable for factor analysis. The result is shown in Table 4.

According to the mode analysis in Table 4, the eight measurement indicators of the campus football development mode are divided into two modes. The first mode belongs to comprehensive method factors, and the second mode belongs to single method factors.

### 3.5. Data Analysis Method

Through the investigation, the campus football data of a university are obtained, and the statistical analysis of Excel and SPSS 17.0 is carried out to analyze the validity and reliability of the questionnaire and the differences between the data of each group so as to fully understand the impact of demographic variables on the development mode of campus football [13]. Firstly, descriptive statistical analysis was performed. Descriptive statistical analysis can preliminaries describe data information, such as output variables and input variables. This paper makes a descriptive statistical analysis of demographic variables, including gender, age, and grade, and takes the percentage as the index [14].

Secondly, validity analysis was performed. Through the factor rotation, the percentage of the factor in the total survey data is obtained and it is tested by KMO measure and Bartle sphere test. Among them, KMO ≥ 0.80 represents significant Bartlett's test. The result is shown in Table 5.

Thirdly, reliability analysis was performed. The Pearson correlation coefficient of the questionnaire distributed in this paper is ≥0.5, which belongs to medium and high reliability and has good content consistency (high efficiency: ≥0.7 Wu [15]; medium validity: 0.5–0.7; low validity: ≤0.3). The result is shown in Table 6.

## 4. Results and Discussion

### 4.1. Sample Selection and Data Source

In this paper, questionnaires were distributed to 13 colleges and universities in area *A*. A total of 420 questionnaires were distributed, and 400 were recovered. The total effective rate was 95.2%, including 10 anonymous questionnaires, 6 questionnaires missing more than 3 answers, and 4 questionnaires with unclear handwriting.

The lowest score of the questionnaire on campus football development mode in this study is 1, and the highest score is 4. Therefore, the middle value of 3 is taken as the reference standard [16].

First, descriptive statistical analysis of demographic characteristic variables, the result is shown in Table 7.

Second, the descriptive statistical analysis of football development model, the result is shown in Table 8.

It can be seen from Table 8 that among the different influencing factors, “football practice form” (3.618) scores higher, indicating that commission and training reward have a great influence on them to stay in the enterprise. The score of “training reward” and “extracurricular practice” are slightly lower, at the middle value of 3, indicating that the incentive index is at the medium level [17]. Thirdly, the influence of demographic characteristic variables on the development model of campus football was assessed. *T*-test and single-factor analysis were carried out to study the influence of gender, age, experience, and grade on the development model of campus football. The result is shown in Table 9.

### 4.2. The Analysis Results

First, gender differences were analyzed, and the result is shown in Table 9. The significant probabilities of campus football development mode, infrastructure, football practice form, practice standard, football match, extracurricular practice, personnel structure, and grade ratio are greater than 0.05, indicating that there is no significant difference in the evaluation of the above indicators between different gender development modes [18]. Second, the age differences are shown in Figure 1.

It can be seen from Tables 3, 4 that students of different ages have significant differences in the variable of football match, but there is no significant difference in other variables.Third, the grade differences is shown in Table 10.

It can be seen from Table 10 that there is no significant difference in the evaluation of students' practice standards, training awards, extracurricular exercises, personnel structure, and grade ratio in different grades.

Fourth, experience differences are shown in Figure 2.

It can be seen from Figure 2 that there is no significant difference in the evaluation of students' practice standards, football matches, training awards, extracurricular exercises, personnel structure, and grade proportion with different experiences.

### 4.3. Effect Analysis

In this paper, Pearson method is used to analyze the relationship between each dimension and the development mode of campus football, and the correlation degree between the indicators is obtained to verify the hypothesis put forward earlier.

First, the correlation analysis of football development model indicators was performed. It can be seen from Table 10 that there is a significant positive correlation between the eight football development model indicators: infrastructure [19], training, football practice forms, football matches, training awards, practice standards, extracurricular practice, personnel structure, and grade ratio, indicating that there is a certain interaction and positive impact among the indicators of football development model. The result is shown in Table 11.

Secondly, correlation analysis between campus football development model and incentive indicators was performed. The result is shown in Table 12.

As shown in Tables 3–8, the comprehensive method factors have the greatest correlation with the football development model, and the correlation coefficient is 0.514. This shows that the comprehensive method factors have a significant positive impact on the development model of campus football. Therefore, the research hypothesis *H*2: Students' comprehensive method has a significant positive impact on the development model of campus football, and the hypothesis is fully established.

### 4.4. Regression Analysis

Taking the development model of campus football as dependent variable and long-term and short-term factors as independent variables, this paper makes a linear retrospective analysis and constructs a regression equation. The analysis results show that the complex correlation coefficient *r* = 0.6443, the judgment coefficient *R*^2^ = 0.235, and the adjusted judgment coefficient *R*^2^ = 0.176, which fully shows that each factor accounts for 64.43% of the total influencing factors, which can explain most of the factors. The result is shown in Table 13.

The analysis results in Table 14 show that the statistical variable *f* = 8.750, and there is a significant correlation between various variables, SIG. < 0.01, indicating that the regression analysis model established in this paper is suitable for the analysis of various indicators, and there is a linear relationship between independent variables (short-term and single-method factors) and dependent variables (football development model) [20], with significant correlation and statistical significance. The result is shown in Table 15.

According to the regression coefficient and test in Table 15, there is a significant correlation between the comprehensive method and the single method in the *t*-test results, and its value is less than 0.01. This shows that the regression coefficient between the two influencing factors is >0.01, and there is a significant correlation. The constant in the regression model is less than 0.01, there is a significant correlation, indicating that there is a significant difference between the constant term and 0.

Through the above analysis results, it can be concluded that the multiple regression equation affecting students' campus football development model is campus football development model = 4.330 + 0.314^*∗*^ comprehensive method factors +0.128^*∗*^ by single method factor formula (4–1). From the regression equation, it can be seen that both comprehensive method factors and single method factors are positive, indicating that these two factors have a significant positive impact on students' football development model. Among them, the influence degree of one method factor (0.314) is the largest, followed by the comprehensive method factor (0.128), and the sig. values of the two variable factors are <0.05, which is statistically significant. This is basically consistent with the above correlation analysis results. Therefore, the development factors of football development model in area a are single, and comprehensive analysis methods should be adopted. The result is shown in Table 14.

From the results of Table 14, we can see that the factors proposed in this paper have a significant impact on the development of campus football, indicating that the research results are reliable. At the same time, the research results of this paper are basically consistent with the related research at home and abroad [21].

## 5. Conclusion

Based on the incentive theory, this paper analyzes the selection of the development mode of campus football, combined with the corresponding theory and the development needs of students [22], puts forward systematic, targeted and different opinions and suggestions so as to ensure the effective development of campus football and give full play to the sports function of campus football. Therefore, the factor analysis method can realize dynamic analysis of multiple factors and improve the accuracy of analysis results. Factor analysis has more obvious advantages and realizes comprehensive analysis of a large number of data. The details are as follows:

1. Local colleges and universities pay more attention to the development mode of campus football and make targeted mode selection according to their own needs, improve students' football enthusiasm, give full play to their own ability, effectively promote the development of campus football and create a good development environment. At the same time, local colleges and universities should aim at the research results of this paper, and put forward measures from the aspects of personnel and system to promote the development of campus football.
2. Colleges and universities should change the concept of campus football model, according to the old concept, combined with students' personal characteristics and needs, give play to the choice of appropriate campus football development model, and promote the corresponding football model development model.
3. Improve the content of football development, build a comprehensive form of campus football development, realize objective and reasonable evaluation, and promote the sustainable development of campus football.

In the process of factor analysis, this paper lacks the comparison between different models. In the future work, we will focus on the comparison between different models.

## Figures and Tables

**Figure 1:** The difference analysis of age on various research variables (*n* = 400).

**Figure 2:** The difference analysis of experience on various research variables (*n* = 400).

**Table 1:** The research assumptions.

Number	Research hypothesis
H_1_	H_1a_ is significant differences in the development model and influencing factors of campus football between different genders
	H_lb_ is significant differences in the development model and influencing factors of campus football at different ages
	H_1c_ is significant differences in the development mode and influencing factors of campus football in different grades
	H_1d_ is significant differences in the development model and influencing factors of campus football with different experience

H_2_	The comprehensive method has a significant positive impact on the development model of campus football

H_3_	The single method has a significant positive impact on the development model of campus football

**Table 2:** The reliability analysis.

Latent variable	Number of variables	Cranach's alpha
Number of variables	8	0.835
Mode 1	2	0.738
Mode 2	6	0.843

**Table 3:** The KMO and Bartlett's test.

Kaiser–Meyer–Olk in measure of sampling adequacy		0.826
Bartlett's test of sphericity	Approx. chi-square	543.983
	df	27
	Sig.	0.000

**Table 4:** The factor analysis results of campus football development model.

Mode code		Load value	Characteristic value	Explanatory ability (%)	Cumulative interpretation (%)
Mode 1	Infrastructure	0.862	2.918	45.9	45.9
	Football practice form	0.746			
	Practice standard	0.744			
	Special salary	0.724			
	Training reward	0.775			
	Extracurricular practice	0.793			

Mode 2	Structure of personnel	0.705	1.023	1.3	64.1
	Grade ratio	0.646			

**Table 5:** The criteria for KMO statistics.

KMO	Suitability of factor analysis
>0.9	Suitability of factor analysis
>0.8	It is very suitable for factor analysis
>0.7	Suitable for factor analysis
>0.6	Factor analysis can be carried out
>0.5	Forced factor analysis
<0.5	Not suitable for factor analysis

**Table 6:** The criteria for reliability coefficient.

Reliability coefficient range	Judgment conclusion
>0.9	Good reliability
0.8-0.9	Good reliability
0.7-0.8	The reliability is average, and some items need to be revised
<0.7	The reliability is not very good. Some items need to be deleted

**Table 7:** The statistics of demographic characteristic variables (*n* = 400).

Demographic variables	Sample distribution	Number (person)	Percentage (%)
	Total number	400	100

Gender	Male	133	33.9
	Female	267	66.1

Age	Under 18	60	15
	18–25 years old	55	13.8
	26–30 years old	35	34.5
	31–35 years old	68	17
	Over 35	85	21.25

Experience	1–5 years	63	15.7
	6–10 years	70	17.6
	11–15 years	83	20.8
	16–20 years	59	14.7

Grade	Secondary specialized school	4	1.0
	Junior college	23	5.8
	Undergraduate	334	83.4
	Master	39	9.9

Grade	Freshman	90	22.4
	Sophomore	220	55.0
	Junior	90	22.7

Experience	A year	54	13.4
	Two years	340	85.0
	More than three years	6	1.6

**Table 8:** The descriptive statistical analysis of football development model indicators (*n* = 400).

Factor	*N*	Maximum	Minimum	Average	Standard deviation
Incentive effect	400	4	1	2.996	0.910
Infrastructure	400	5	1	2.866	0.849
Football practice form	400	5	1	3.618	0.747
Practice standard	400	5	1	3.161	0.654
Football match	400	4	1	2.882	0.851
Training reward	400	5	1	3.616	0.745
Extracurricular practice	400	5	2	2.995	0.63
Structure of personnel	400	5	1	3.163	0.911
Grade ratio	400	5	2	2.872	0.851

**Table 9:** The difference analysis of gender on various research variables (*n* = 400).

Research variables	Gender	*N*	Mean value	Standard deviation	*T* value	Sig.
Development model of campus football infrastructure	Male	133	3.44	0.821	0.977	0.779
	Female	267	3.91	0.905		

Football practice form practice standard	Male	133^*∗*^	3.06	0.908	0.928	0.753
	Female	267	2.94	0.880		

Football match training reward	Male	133	3.88	1.328	0.598	0.074
	Female	267	3.76	1.495		

Extracurricular practice structure of personnel	Male	133	3.80	0.896^*∗*^	−0.059	0.130
	Female	267	3.80	0.999		

Grade ratio research variables	Male	133	3.42	0.789^*∗*^	1.248	0.264
	Female	267	3.27	0.917		

Development model of campus football infrastructure	Male	133	3.57	0.879^*∗*^	−0.733	0.034
	Female	267	3.79	1.031		

Football practice form practice standard	Male	133	3.59	0.829^*∗*^	−0.592^*∗*^	0.390
	Female	267	3.66	0.892		

Football match training reward	Male	133	3.52	0.803	1.103	0.578^*∗*^
	Male	267	3.39	0.843		

Extracurricular practice	Female	133	3.21	0.738
	Male	267	3.17	0.699	0.399	0.289^*∗*^

^*∗*^ *P* < 0.05.

**Table 10:** The analysis on the differences of various research variables in grade.

	Secondary specialized school	Junior college	Undergraduate	Master	*F*	Sig.
Incentive effect	2.26	2.79	3.24	3.02	3.775	0.027
Infrastructure	2.55	2.81	2.91	3.33	4.311	0.001
Football practice form	3.73	3.76	3.55	3.89	1.284	0.015
Practice standard	3.18	3.39	3.57	3.86	3.363	0.092
Football match	3.45	3.17	3.19	3.58	3.486	0.795
Training reward	3.55	3.60	3.64	3.94	4.227	0.331
Extracurricular practice	3.27	3.35	3.66	3.89	^*∗*^976	0.351
Structure of personnel	2.73	2.97	3.43	3.83	7.311	0.255
Grade ratio	3.18	3.05	3.02	3.36	3.507	0.102

**Table 11:** Correlation analysis results of football development model indicators (*n* = 400).

	*x*_1_	*x*_2_	*x*_3_	*x*_4_	*x*_5_	*x*_6_	*x*_7_	*x*_8_
*x*_1_								
*x*_2_	0.182^*∗∗*^							
*x*_3_	0.115	0.014	1					
*x*_4_	0.259^*∗∗*^	0.094	0.129	1				
*x*_5_	0.307^*∗∗*^	0.121^*∗*^	0.203^*∗∗*^	0.556^*∗∗*^	1			
*x*_6_	0.389^*∗∗*^	0.105	0.078	0.553^*∗∗*^	0.605^*∗∗*^	1		
*x*_7_	0.194″	0.126	0.215^*∗∗*^	0.257^*∗∗*^	0.251^*∗∗*^	0.266^*∗∗*^	1	
*X*_8_	262^*∗*^	0.072	0.133	311^*∗∗*^	0.365^*∗∗*^	0.497^*∗∗*^	0.127	1
*N*	400	400	400	400	400	400	400	400

^*∗∗*^Significantly correlated at the 0.01 level (bilateral);^*∗*^Significant correlation at 0.05 level (bilateral). *X*_1_ = infrastructure, *X*_2_ = football practice form, *X*_3_ = football match, *X*_4_ = training reward, *X*_5_ = practice standard, *X*_6_ = extracurricular practice, *X*_7_ = personnel structure, *X*_8_ = grade proportion.

**Table 12:** The correlation analysis results between campus football development model and various indicators.

	Pearsonrelevance	0.514^*∗∗*^
Single method factor		
	Significance (bilateral)	0.000
	Pearson relevance	0.47^*∗∗*^

Comprehensive method factors		
	Significance (bilateral)	0.000
*N*	400	

^*∗∗*^Significantly correlated at the 0.01 level (bilateral).

**Table 13:** The model summary.

Model summary				
Model	*R*	*R* ^2^ adjustment	*R* ^2^ standard	Standard
1	0.469a	0.235	0.176	0.34962

Predictive variables (constant): comprehensive method factors and single method factors. Dependent variable: football development model.

**Table 14:** The regression coefficient and test.

	*B*	Standard error	Standardized coefficient	*T*	Sig.
Constant	4.330	0.036		2.458	0.000
Comprehensive method	0.314	0.036	0.432	8.025	0.000
Single method	0.128	0.036	0.378	5.907	0.000

Dependent variable: development model of campus football.

**Table 15:** The analysis of variance results.

Model	Sum of squares	df	Mean square	Sig.
Regression	20.077	5	4.0158.750	0.000^a^
Residual	27.381	224	0.122	
Total	47.458	229		

Predictive variable (constant): comprehensive method and single method; Dependent variable: development model of campus football.

## Data Availability

The data used to support the ﬁndings of this study are available from the corresponding author upon request.
